# The Correlation between Children's Intelligence Quotient and Their Behavior in Dental Setting: A Cross-Sectional Study

**DOI:** 10.1155/2022/2299215

**Published:** 2022-06-24

**Authors:** M. Khosrozadeh, S. Ghadimi, M. Kazemzadeh Gharghabi, M. J. Kharrazifard, M. H. Hamrah, A. Baghalian

**Affiliations:** ^1^Department of Pediatric Dentistry, School of Dentistry, Tehran University of Medical Sciences, Tehran, Iran; ^2^Dental Research Center, Tehran University of Medical Sciences, Tehran, Iran

## Abstract

Children with high intelligence quotient (IQ) are more capable of managing adverse situations. These children may show more cooperation to receive dental treatments. This study assessed the effect of intelligence quotient (IQ) of 5-10-year-old children on their cooperation during dental treatments. Eighty children without previous dental history and in need of pulpotomy and stainless steel crowns in one tooth were selected. A written consent was obtained from the parents, and after the children's IQ was measured by Raven intelligence test, the treatments were performed and their cooperation level was determined using Frankl's behavior rating scale with rating 1 to rating 4 (definitely negative, negative, positive, and definitely positive). In this cross-sectional study, the relationship between IQ and cooperation level was analyzed by one-way ANOVA test while the effect of age and gender on IQ and cooperation level was studied by ordinal regression test. Out of the total samples, 5% had definitely negative, 16.2% had negative, 56.3% had positive, and 22.5% had definitely positive level of cooperation according to Frankl criteria. There was a significant and positive correlation between IQ and level of cooperation (*r* = 0.87, *p* < 0.001). According to the results of the linear regression analysis, to examine the effect of age, sex, and IQ variables on cooperation, children's age (*p* value = 0.003) had a positive effect on their cooperation, but gender had no effect on predicting IQ and cooperation level (*p* value = 0.557). Regarding significant relationship between IQ scores and cooperation level, dentists can predict cooperation in pediatric patients to deliver better treatments and increase patients' satisfaction.

## 1. Introduction

Dental appointment can cause the patient to experience serious fear and discomfort and lead to some certain unpredictable responses which might be followed by decreased acceptance of dental treatment [1, 2]. Childhood dental fear/dental behavior management problems (BMP) are categorized as multifactorial issues with vastly various underlying explanations such as differences in child rearing, personality traits, the child's sociocultural background, parental experience, and particularly anxiety. Cognitive and social adaptive skills and the ability to learn strategies for coping with stressful and routine conditions may alter the child's response to dental environment [1, 3, 4].

Anxiety might boost sensory receptivity and pain perception and exacerbate the situation for the child's cooperation [5, 6]. Dental anxiety is considered to be the fifth most commonly feared situation; however, it is expected to reduce with age [7].

Dentistry as an interactive field has put more and more emphasis on the human dimension of the relationship between dental practitioners and patients. Although technology has made great improvements in dentistry nowadays, our task as a pediatric dentist is still the same: to carry out dental procedures on children with variant ranges of cooperation [8]. According to Wright et al., as a dental health team, we are supposed to follow two main goals: to perform an effective and efficient dental treatment and to initiate positive attitude in the patients [9]. Not only the patients' overall physical condition but also their psychological and mental state should be of great concern to the caregiver [10].

As defined by Raven's Progressive Matrices, intelligence is believed to be a general skill, termed *fluid ability* or *fluid intelligence* versus acquired knowledge or *crystallized intelligence*.

Fluid intelligence is often used interchangeably with reasoning ability in the current context.

Per se, it is not a static characteristic of human behavior, and a variety of maturational and experiential elements can influence fluid intelligence [11–13].

Intelligence quotient (IQ) is defined as the relative intelligence of an individual recorded as a score on a standardized test of intelligence, which will influence the child's understanding of causes and consequences, information, and instructions [14] and also influence their behavior and feedback in the dental setting [15].

It is believed that intelligence quotient can be a strong predictor of an individual's success in all features of life as the general index of cognitive ability [1]. Many studies have found an association between low intelligence and psychological disorders during childhood [16, 17].

General intelligence is proven to have more significant impact on a child's anxiety in his first dental visit [10]. A preceding study showed that it took a considerably longer time for children of low IQ (<68) to accept dental treatment [18].

In children with intellectual disability, the situation may become more complicated, and there seems to be a serious gap in the knowledge dealing with these patients and their behavioral conditions. People with considerably low intellectual capacity and adaptive behavior might suffer significant problems in everyday life. Intellectual impairment, like intellectual ability, appears on a continuum and must be characterized and understood in this way. Individuals with intellectual disabilities, regardless of their diagnostic test scores, require assistance tailored to their specific needs and preferences [19].

In this study, it was aimed to investigate whether children's IQ levels are related to their performance during dental treatment and the relationship between IQ and children's cooperation. The impact of this issue on the type and quality of their behavior in dental settings will be scrutinized.

Apparently, few studies have been conducted in pediatric patients focusing on the effect of children's intelligence on their behavior in medical settings. Nevertheless, the achievements of these studies can be advantageous on common behavior control techniques and management of young patients in terms of estimating their level of cooperation.

## 2. Materials and Methods

In this observational cross-sectional study, eighty healthy children (47 girls and 33 boys) aged 5 to 10 years old were considered. They were selected from new patients referring to the Department of Pediatric Dentistry, Tehran University of Medical Sciences, Tehran, Iran, within the period from December 2019 to July 2020.

This study was approved by the ethical committee of Tehran University of Medical Sciences (IR.TUMS.DENTISTRY.REC.1398.175) and was conducted in adherence to the Declaration of Helsinki. Eligibility for the study was assigned according to the following criteria:

- Physical and mental health of children
- No previous experience of dental treatment
- No history of unpleasant experience in a medical setting
- At least one carious primary molar in need of pulpotomy and stainless steel crown treatment

And those with criteria in contrary to those mentioned above and also the patients whose treatment session lingers more than 30 minutes were excluded from the study.

During the first visit, the child was thoroughly examined by a pediatric dentist, necessary radiographs were obtained, and those who had at least one primary molar in need of pulpotomy and stainless steel crown treatment were considered for the study. Each child also received oral prophylaxis in the first session in order to become acquainted to the dental setting. After explaining the procedure and objectives of the study to the parents, their informed written consents were taken.

Raven's Progressive Matrices (RPM) for IQ measurement were used. Since these matrices are designed for children 5 to 11 years old, the similar age group was selected for the study.

The data required for this study were collected in two consecutive sessions for each child. In the first session, before enrolment, an IQ test with RPM was performed in an environment other than the dental treatment site, and the second session was scheduled for the aforementioned specific dental intervention. The child's behavior was assessed according to Frankl's scale. Parents were not present during either of these sessions. In this way, the interference with the behavior of the child and the dentist during the work was eliminated. This seems to prevent them from transmitting their stress to the child and distracting him. This was stated in the informed consent.

To avoid any interference and distraction, only one subject was tested each time. In order to make children feel more comfortable during the test, the administrator conducted RPM in a serene atmosphere far from the dental setting in ~15-20 minutes. The pediatric dentist who conducted the treatment was supposed to evaluate the child's behavior according to Frankl's scale at the end of the appointment and was not aware of the result of the IQ test taken at the first visit. After the initial visit, a second session was set to perform the treatment and evaluate the child's behavior during the procedure. Children were prepared for the treatment by using the Tell-Show-Do (TSD) technique; then, local anesthetic (lidocaine 2%; epinephrine 1/100000; short needle; gauge 27) (Darou Pakhsh, Tehran, Iran) was injected slowly following the application of topical anesthetic gel (benzocaine 5%). After waiting for 5 minutes to make sure about the depth of anesthesia, a five-minute formocresol pulpotomy and classic stainless steel crown preparation was performed by the pediatric dentist who was blind to the results of RPM.

The child's behavior was assessed according to Frankl's behavior rating scale, ranging from 1 to 4 (Table 1) with “1” being definitely negative and “4” definitely positive behavior and attitude [20]. Thus, in this study, children were divided into 4 separate groups based on Frankl's behavioral scale and were carefully examined.

In order to eliminate the effect of age on child behavior, it was tried that the number of cooperative and uncooperative children in different age groups be equal.

Participants were not divided into groups according to IQ levels. An IQ score was recorded, and the behavior was analyzed based on the IQ rate.

The formula for determining the sample size was applied using the correlation coefficient. Based on the results of the pilot study, considering the *α* = 0.05 and 80% power to evaluate 4 variables, and the value of *R* = 0.1, the minimum required sample size of 113 people was estimated, but according to the onset of coronavirus at the time of this study and the pandemic of the virus worldwide, after consulting a statistical expert, the sample size was reduced to 80.

The correlation between intelligence quotient and Frankl's behavior rating scale was statistically investigated according to the one-way ANOVA test.

Considering the dispersion of IQ variances in different levels of cooperation (Levene test; *p* value = 0.001), Dunnett's multiple comparison post hoc test was used for pair-wise comparison.

The ordinal regression model was applied to determine the simultaneous effect of age, gender, and IQ on the children's cooperation. Obtained data was analyzed using SPSS 25.0 version (SPSS for Windows; SPSS Inc., Chicago, IL) with the statistical type I error (*α*) being 0.05.

## 3. Results

Eighty children (47 girls and 33 boys) with the mean age of 7.25 ranging from 5 to 10 years old were investigated. Mean IQ and SD according to the Frankl scale is shown in Table 2.

Mean IQ (SD) in group 1 (4 children) with definitely negative cooperation was 73.50 (3.000), in group 2 (13 children) with negative cooperation was 85.92 (6.062), in group 3 (45 children) with positive cooperation was 100.40 (6.890), and in group 4 (18 children) with definitely positive cooperation was 114.83 (16.843).

The mean IQ score (SD) for all participants was 99.95 (14.553).

Homogeneity of variance of different groups was evaluated based on the Levene test. Analysis of variance or ANOVA test is one of the statistical models that can examine the differences between groups or categories.  Table 3 demonstrates the results of the one-way ANOVA test of IQ levels in different cooperation levels according to Frankl's behavior scale. As summarized in Table 4, according to the ANOVA test, there is a significant difference in the amount of IQ between four groups of cooperation. Considering the dispersion of IQ variances in different levels (Levene test; *p* value = 0.001), Dunnett's multiple comparison post hoc test was used for pair-wise comparison.

In the analysis of variance, if the null hypothesis is excluded (if the difference is significant), post hoc tests could be used to detect differences within groups, in fact, to see which of these groups has this difference (Table 4).

Table 5 depicts the results of the ordinal regression test and shows that the children's age and intelligence quotient have a significant role in their cooperation.

## 4. Discussion

This study was designed to investigate the impact of children's IQ on their behavior and the relationship between intelligence and cooperation in the dental setting. In the current research, a significant and positive correlation was found between IQ and children's cooperation according to Frankl's scale.

Since Raven's test is widely used in Iran and its subset of progressive matrices is designed for children 5 to 11 years old and people with physical and mental disabilities, Raven's Progressive Matrices (RPM) for IQ measurement were used [21].

Children with low IQ need significantly longer time to accept the dental treatment situation. Children with above-average IQ had positive levels of cooperation, and those with superior IQ had definitely positive cooperation during the dental procedure. On the other hand, children with borderline IQ seemed to have negative cooperation, and those with below-average IQ had definitely negative cooperation. That is to say, as the children's intelligence quotient increases, so does their level of cooperation, and they tend to exhibit better and more constructive communication and cooperation. This helps the child to have an efficient predominance over his stress and anxiety [1, 22].

Intelligence and sensory processing seem to be closely related; hence, intelligent children show higher speed of sensory processing. Both visual and auditory processing have a critical role in intelligence. However, considering pediatric patients, auditory stimuli tend to be less restrictive. An et al. found a positive correlation between the intelligence quotient and percent change of gamma increase relative to baseline in the auditory cortex [23]. The results of this study are in line with the current study's findings. Verbal distraction as a behavior management technique is the main method during dental treatment of pediatric patients, and as the present study suggests, in children with higher levels of IQ, a higher pace of auditory information processing and better cooperation are expected.

In a study to determine predictive factors for children behavior in the dental environment, the majority of children demonstrated cooperative attitude. The child's age, the technique employed, and the expertise of the dental practitioner may be the potential reasons for this result. Many children have adequate cognitive capacity after four years of age to control their fear and comply with dental treatment. In this study, 13.7% of children assumed to be extremely anxious presented promising behavior. Since it is especially designed for preschool children and also has moderate to high reliability in distinguishing anxious and nonanxious children, the Venham picture test (VPT) was used in the study. Three predictive variables were correlated with child behavior in the aforementioned study: the mother's estimation of the child's behavior, the level of anxiety of the child (VPT), and whether the child had suffered from a toothache before [24].

In accordance with this study, Shetty et al. found a significant positive correlation between IQ and Frankl's behavior scale in healthy children while no correlation in the group with hearing and speech impairment was recorded [15]. Considering that in this study, the Culture Fair Intelligence Test Scale 3 (CFIT) and performance scale (nonverbal) were used to measure IQ, and also due to the limitations caused by the existence of speech and hearing impairments for the correct implementation of behavior management, especially Tell-Show-Do (TSD), this difference in results is justifiable.

Unlike the current study, Aminabadi et al. reported no correlation between the IQ and child's cooperation in a group of healthy patients, although a significant negative correlation between children's behavior and total EQ (Emotional Quotient) score was observed [1]. It seems that performing two different dental interventions in two studies (pulpotomy and stainless steel crown versus class II amalgam restoration) as well as using sound, eye, and motor (SEM) and modified child dental anxiety scale (MCDAS) criteria to assess the child's behavior and anxiety during treatment can explain this difference in results.

It is worth mentioning that this cross-sectional study presents results of data collected from a convenience sample, which limits its external validity. Therefore, these findings should be interpreted and discussed with this limitation in mind. There is a lack of a longitudinal study in the literature involving randomly selected representative samples that present more consistent scientific evidence regarding the assessment of child behavior in the dental setting. In addition, most of the patients attending in the study are from the average socioeconomic class which can be a confounding factor in this research since it is well-known that there is a significant correlation between socioeconomic status and IQ [25].

On the other hand, the limited facilities of the research center in comparison with its private counterparts do not allow the creation of an ideal atmosphere that is compatible with child psychology, and this issue can also adversely affect the outcome of the research.

It is also interesting to study the cooperation of children with different IQ levels during different medical and dental interventions.

## 5. Conclusion

High IQ in children paves the way for them to cope better with the new and unfamiliar dental environment. To look at the issue optimistically, the results of IQ assessment with similar pretreatment methods can be generalized to the findings of this study. The results of this study showed that knowing the level of IQ in children can also help dentists in deciding to treat them in routine dental office conditions or choosing treatments under general anesthesia.

## Figures and Tables

**Table 1:** Frankl's classification (Frankl's behavior rating scale 1962).

Rating	Attitude	Definition
1	Definitely negative	Refusal of treatment, crying forcefully, fearful, or any other overt evidence of extreme negativism
2	Negative	Reluctant to accept treatment, uncooperative, some evidence of negative attitude but not pronounced, i.e., sullen and withdrawn
3	Positive	Acceptance of treatment; at times curious, willingness to comply with dentist, at times with reservation but patient follows the dentist's directions cooperatively
4	Definitely positive	Good rapport with the dentist, interested in the dental procedures, and laughing and enjoying the situation

**Table 2:** Descriptive values (mean, standard deviation, standard error, minimum, and maximum) of IQ and cooperation according to Frankl's behavior scale.

Cooperation	No. of patients	Mean IQ	Std. deviation	Std. error	95% CI		Min.	Max.
					Lower bounds	Upper bounds		
1	4	73.50	3.000	1.500	68.73	78.27	72	78
2	13	85.92	6.062	1.681	82.26	89.59	78	100
3	45	100.40	6.890	1.027	98.33	102.47	91	118
4	18	114.83	16.843	3.970	106.46	123.21	83	146
Total	80	99.95	14.553	1.627	96.71	103.19	72	146

**Table 3:** Results of the one-way ANOVA test of IQ levels in different cooperation levels according to Frankl's behavior scale.

	Total squares	Df	Mean square	*F*	*p* value
Intergroup	9352.577	3	3117.526	32.108	0.001>
Intragroup	7379.223	76	97.095		
Total	16731.800	79			

**Table 4:** Results of Dunnett's multiple comparison post hoc test of IQ levels in different cooperation levels according to Frankl's behavior scale.

Compared groups		Mean difference	Std. error	*p* value	95% CI	
					Lower bounds	Upper bounds
1	2	-12.423^∗^	2.253	0.001	-19.63	-5.22
	3	-26.900^∗^	1.818	0.001>	-33.72	-20.08
	4	-41.333^∗^	4.244	0.001>	-53.72	-28.95

2	1	12.423^∗^	2.253	0.001	5.22	19.63
	3	-14.477^∗^	1.970	0.001>	-20.17	-8.78
	4	-28.910^∗^	4.311	0.001>	-41.33	-16.49

3	1	26.900^∗^	1.818	0.001>	20.08	33.72
	2	14.477^∗^	1.970	0.001>	8.78	20.17
	4	-14.433^∗^	4.101	0.013	-26.44	-2.42

4	1	41.333^∗^	4.244	0.001>	28.95	53.72
	2	28.910^∗^	4.311	0.001>	16.49	41.33
	3	14.433^∗^	4.101	0.013	2.42	26.44

**Table 5:** Results of ordinal regression analysis to investigate the effect of age, gender, and IQ on the cooperation.

Independent factor	Standardized coefficients			*t*	*p* value
	*B*	Std. error	Beta		
Age	0.110	0.035	0.225	3.091	0.003
Gender	0.066	0.112	0.043	0.590	0.557
IQ	0.041	0.004	0.777	10.711	0.001>

∗The mean difference is significant at 0.05.

## Data Availability

The raw data supporting results of this article would be available upon request from the corresponding author.

## References

[1] Aminabadi N. A., Erfanparast L., Adhami Z. E., Maljaii E., Ranjbar F., Jamali Z. (2011). The impact of emotional intelligence and intelligence quotient (IQ) on child anxiety and behavior in the dental setting. *Acta Odontologica Scandinavica*.

[2] Guinot Jimeno F., Mercadé Bellido M., Cuadros Fernández C., Ai L. R., Llopis-Perez J., Quesada B. (2014). Effect of audiovisual distraction on children's behaviour, anxiety and pain in the dental setting. *European Journal of Paediatric Dentistry*.

[3] Arnrup K., Broberg A. G., Berggren U., Bodin L. (2002). Lack of cooperation in pediatric dentistry-the role of child personality characteristics. *Pediatric Dentistry*.

[4] Majstorovic M., Morse D. E., Do D., Lim L., Herman N. G., Moursi A. M. (2014). Indicators of dental anxiety in children just prior to treatment. *The Journal of Clinical Pediatric Dentistry*.

[5] Aminabadi N. A., Pourkazemi M., Babapour J., Oskouei S. G. (2012). The impact of maternal emotional intelligence and parenting style on child anxiety and behavior in the dental setting. *Medicina Oral, Patologia Oral y Cirugia Bucal*.

[6] Erfanparast L., Vafaei A., Sohrabi A. (2015). Impact of self-concept on preschoolers' dental anxiety and behavior. *Journal of Dental Research, Dental Clinics, Dental Prospects*.

[7] Hmud R., Walsh L. J. (2007). Dental anxiety: causes, complications and management approaches. *International Dentistry SA Australasian Edition*.

[8] Sheller B. (2004). Challenges of managing child behavior in the 21st century dental setting. *Pediatric Dentistry*.

[9] Wright G. Z., Starkey P. E., Gardner D. E. (1983). Managing children’s behavior in the dental office. *Mosby*.

[10] Toledano M., Osorio R., Aguilera F. S., Pegalajar J. (1995). Children's dental anxiety: influence of personality and intelligence factors. *International Journal of Paediatric Dentistry*.

[11] Fry A. F., Hale S. (2000). Relationships among processing speed, working memory, and fluid intelligence in children. *Biological Psychology*.

[12] Carpenter P. A., Just M. A., Shell P. (1990). What one intelligence test measures: a theoretical account of the processing in the Raven progressive matrices test. *Psychological Review*.

[13] Horn J. L., Cattell R. B. (1967). Age differences in fluid and crystallized intelligence. *Acta Psychologica*.

[14] Psychological index terms via unified medical language system at the National Library of Medicine. http://nlm.nih.gov/glossary=intelligencequotient.

[15] Shetty R. M., Pashine A., Jose N. A., Mantha S. (2018). Role of intelligence quotient (IQ) on anxiety and behavior in children with hearing and speech impairment. *Special Care in Dentistry*.

[16] Greenberg M. T., Kusche C. A., Cook E. T., Quamma J. P. (1995). Promoting emotional competence in school-aged children: the effects of the PATHS curriculum. *Development and Psychopathology*.

[17] Anderson J., Williams S., McGee R., Silva P. (1989). Cognitive and social correlates of DSM-III disorders in preadolescent children. *Journal of the American Academy of Child & Adolescent Psychiatry*.

[18] Rud B., Kisling E. (1973). The influence of mental development on children's acceptance of dental treatment. *European Journal of Oral Sciences*.

[19] Snell M. E., Luckasson R., Borthwick-Duffy W. S. (2009). Characteristics and needs of people with intellectual disability who have higher IQs. *Intellectual and Developmental Disabilities*.

[20] Frankl S. S. F., Fogels H. (1962). Should the parent remain with the child in the dental operatory. *Journal of Dentistry for Children*.

[21] Raven J. (2000). The Raven's progressive matrices: change and stability over culture and time. *Cognitive Psychology*.

[22] Olszewski A. K., Radoeva P. D., Fremont W., Kates W. R., Antshel K. M. (2014). Is child intelligence associated with parent and sibling intelligence in individuals with developmental disorders? An investigation in youth with 22q11.2 deletion (velo-cardio-facial) syndrome. *Research in Developmental Disabilities*.

[23] An K. M., Hasegawa C., Hirosawa T. (2020). Brain responses to human-voice processing predict child development and intelligence. *Human Brain Mapping*.

[24] Ramos-Jorge M. L. M. L., Pavia S. M., Serra-Negra J. M., Pordeus I. A. (2006). Predictive factors for child behaviour in the dental environment. *European Archives of Paediatric Dentistry*.

[25] Von Stumm S., Plomin R. (2015). Socioeconomic status and the growth of intelligence from infancy through adolescence. *Intelligence*.

